# Multimodal English Teaching Classroom Interaction Based on Artificial Neural Network

This article has been retracted.

**DOI:** 10.1155/2022/3141451

**Published:** 2022-05-28

**Authors:** Wenbin Hua

**Affiliations:** School of Foreign Languages, Hubei University of Arts and Science, Xiangyang 441000, Hubei, China

## Abstract

In recent years, with the rapid development of science and technology, traditional teaching methods and concepts have been frequently impacted. Artificial neural network shows excellent intelligence because of its powerful nonlinear processing ability and efficient associative function. It is increasingly becoming an emerging object in the field of artificial intelligence. At the same time, in the field of education and teaching, the integration of English teaching and multimodality not only condenses the characteristics of the times but also expands new teaching models, bringing opportunities for the emergence of new teaching models. Based on this, this study proposes an interactive method for multimodal English teaching based on artificial neural networks. It aims to study how to use the autonomous learning of artificial neural networks to accelerate the fusion of different modalities and at the same time make suggestions for different teaching interaction modes. This paper firstly analyzes the interaction of English teaching under the traditional mode. It then proposes a multimodal fusion interaction method based on artificial neural networks. It finally explores the feasibility of the new interaction theory by setting up an experimental group and a control group. Through the analysis of the experimental data, the final data results show that the multimodal fusion interaction based on artificial neural network has a very significant effect, and the students' interest in the English classroom is as high as 81.9%. This fully demonstrates the great value of the new fusion method, and it has certain enlightening significance for the establishment of English teaching modes and curriculum reform.

## 1. Introduction

In the school environment, the classroom is the first scene where students acquire knowledge and grow. However, in years of teaching practice and experience summarization, it has been found that the level of classroom interaction will also have an important impact on the acquisition of knowledge. In particular, the English classroom has brought great inconvenience to the interaction of the English teaching classroom because of the particularity of the language and the influence of noncommunication. On the one hand, students' acceptance of multimodal teaching is different, which reduces the overall process and efficiency of teaching. On the other hand, despite the introduction of new modalities of teaching, the difficulty of the English subject itself has not decreased, so the original problems faced by students have not been solved.

Therefore, this paper focuses on the research and analysis of how to make full use of the characteristics of the English subject, so that students can have immersive learning. At the same time, this paper also combines artificial neural networks to design learning methods suitable for each type of students through prediction and learning methods, so that students can truly learn happily. The multimodal teaching interaction model based on artificial neural network can change the English classroom from boring to joyful. In this classroom environment, students can get rid of the traditional passive learning state in one fell swoop, thus transforming into a positive self-learning attitude. This can not only improve students' comprehensive English literacy but also further cultivate outstanding students with good character and personality.

The innovations of this paper are as follows:

1. This paper cleverly combines artificial neural networks with multimodality. It proposes an interactive mode of English teaching based on the integration of the two, which is of great significance to the integration of educational resources and the reform of teaching methods in the new era.
2. This paper integrates theories of natural science, education, and information science. On this basis, a multimodal teaching interaction method based on artificial neural network is produced, which greatly improves the overall participation in classroom teaching.

## 2. Related Work

Alanis used the well-known Lyapunov method for scaling artificial neural networks trained by Kalman filter-based algorithms. At the same time, he used a one-step ahead and an n-step ahead of the European power system data. He presented the results of using a recurrent neural network training algorithm based on the extended Kalman filter and its application in electricity price forecasting [1].

Santosh presented a study of various artificial neural network (ANN) algorithms to select the most appropriate algorithm for diagnosing transients in a typical nuclear power plant (NPP). By conducting optimization research on several neural network algorithms, he developed a neural network-based framework. It is designed to help operators quickly identify such initial events and take corrective actions [2].

Hodo started with the threat analysis of IoT. He focused on the classification of normal and threat patterns on IoT networks and introduced artificial neural networks (ANNs) to address these threats. He first validated a simulated IoT network and then trained it using Internet packet tracing with a multilevel perceptron and then evaluated its ability to block distributed denial of service (DDoS/DoS) attacks [3].

Safa employed an artificial neural network (ANN) approach for simulating wheat production. He estimated average wheat yields based on extensive data collection involving 40 farms in Canterbury, New Zealand, and eventually developed computational models based on artificial neural networks. Based on this, the model can predict wheat yield under different conditions and farming systems using direct and indirect technical factors [4].

Kjaerg Aard pointed out that, with the advent of Web 2.0, multimodal teaching has become a popular literacy practice. However, the potential of multimodality in education is currently underexploited. He examined how multimodality positively impacts reading and writing in a case study of 150 teachers' teaching, with a focus on multimodal teaching in primary and secondary school settings [5].

Yun-Hee pointed out that the multimodal form of classroom interaction can improve classroom satisfaction. However, most studies tend to look at it from a cognitive perspective. To study the classroom interaction satisfaction model, he used LISREL structural modeling. He proposed survey studies to test hypotheses concerning faculty presence, student interaction, PAD, and satisfaction and collected student data involving one university [6].

To solve the problem of imbalanced data distribution and improve the prediction performance of protein-metal-ion interaction sites (PMIIS), Qiao L proposed a novel class-imbalanced learning algorithm combining undersampling and oversampling methods. He also designed a new sequence-based prediction method based on a new class-imbalanced learning algorithm and a support vector machine (SVM) algorithm. He also constructed a relatively complete standard dataset [7].

## 3. Classroom Interaction of Multimodal English Teaching Based on Artificial Neural Network

### 3.1. Artificial Neural Network

Artificial neural network is a major research hotspot in the field of artificial intelligence. It covers a wide range of fields and directions. It can be seen in many popular fields, such as economic forecasting, market environment forecasting, benefit monitoring, and intelligent image recognition. We will introduce its composition, working principle, and application fields one by one [8].

#### 3.1.1. Neurons

To understand the neural network, it is necessary to go back to the neuron cell [9]. In the field of biology, neurons are the basic structural and functional units of information processing in the nervous system. We all know that the general biological neurons are mainly composed of dendrites, axons, synapses, and cell bodies. In artificial neural networks, people also derive corresponding functional divisions by simulating biological neurons. In an artificial neural network, the artificial neuron is its basic information processing unit. A simple neuron structure is shown in Figure 1.

It can be seen from Figure 1 that a neuron is a multielement input and single-element output structure. This structure is a nonlinear functional element. It consists of input variables, weights, accumulation function, activation functions, and output values.

#### 3.1.2. Neural Networks

After talking about neurons, let us look at what a neural network is [10]. In regard to this, people's first reaction is the nerve cells in the organism's brain. It is reported that there are 14 billion neuron cells in the human brain, and its complexity is no less than the structure of network nodes. The artificial neural network is actually a set of biomimetic models established by people imitating biological neurons. To generalize it to other fields, the neural system is mathematicized and closely linked to the field of artificial intelligence, resulting in artificial neural networks. This is shown in Figure 2 [11].

#### 3.1.3. Characteristics of Artificial Neural Network

Artificial neural network has unparalleled advantages and characteristics. The following aspects will be elaborated.

First, the ability is to learn independently. Artificial neural network is a biological neural network that simulates autonomously, so its first feature is self-learning ability [12]. Organisms can process information billions of times through neurons, evolving themselves in the process. They are placed in the artificial neural network, and the computer can also learn and train autonomously and continuously improve the processing efficiency in the process. For example, in the intelligent recognition of images, we only need to put the set of images to be recognized and the corresponding recognition results into the neural network, which can continuously realize the intelligent recognition of images through self-learning. With the continuous increase of training samples and the continuous passage of time, its recognition accuracy and speed will increase exponentially.

Second, it has Lenovo storage capabilities. The continuous development of artificial nerves has led to other neural networks. Among them, the feedback neural network can use association to store data and information [13]. In this way, in the face of large data information, the network can realize storage and calling through the association between data. This not only saves the storage space but also effectively improves the calling speed of data. In this storage process, the neural network can also continuously optimize and upgrade through autonomous learning, to find the optimal storage solution for each stored process.

Third is the ability to find the optimal solution at high speed. The process of finding the optimal storage solution can actually be regarded as an example of finding the optimal solution. Because there are often many solutions to a complex problem and, in this process, there is often only one solution that is optimal, the process of continuously obtaining the optimal solution often requires strong computing power support. On this issue, the advantages based on neural networks are vividly displayed and, coupled with their autonomous learning ability and effective storage, neural networks have a double blessing in dealing with large-scale problems.

#### 3.1.4. Artificial Neural Networks and Education

Artificial neural networks continue to develop, so their connections to other fields are getting closer [14]. A dynamic video or image is a great opportunity for interaction. Teachers can select the films in the English classroom, so that they know what to do. They choose video materials that are appropriate to the student's English level and fit the topic. They introduced foreign language film and television works of the same theme to students and guided them to discuss and think. While watching the film, students can learn authentic spoken English. Foreign language learning software is a good way to help. The computer can adjust the difficulty level of the test questions according to the student's test level. This can not only show students dynamic topics but also automatically generate analysis sheets and test scores. In the field of artificial intelligence, its integration with applications such as intelligent image recognition and speech recognition is accelerating. In the field of education, its powerful characteristics also quickly found a foothold for it. In the information interaction with multiple modalities, the neural network is endowed with a new modal fusion theory. Its main application areas are shown in Figure 3 [15].

### 3.2. Multimodal Theory

#### 3.2.1. Social Symbols

Social symbols, as the name suggests, are various symbols in social life. They mainly include language and culture. Semiotics was born relatively early. It can be traced back to ancient Greece, although it has a long history. However, it was not until the middle of the last century that semiotics officially became a discipline, an independent discipline [16]. The reason is that the development of science and technology has provided large technical support for the qualitativeness and quantification of social symbols. After the development of social semiotics, a relatively complete system has been established. These include studies of language, sound, and images. In the process of its continuous development, the focus of social symbols gradually penetrated into the multimedia field and further influenced the development of the media field. The main application field of multimedia, pedagogy, has also become the next target. The multimodal teaching theory based on social semiotics has directly influenced the traditional teaching mode.

#### 3.2.2. System Functional Language

On the basis of semiotics, people began to work on a systematic linguistic theory [17]. Because, under the background of traditional semiotics, language and writing are all isolated symbols, which do not form a complete system, it is widely believed that language forms the crux of the entire system of symbols, because language is generally used to express related information. Therefore, people decide to build a system network on this basis and want to build a functional language system with language communication as the carrier. Under this trend of thought, people have further discovered the information elements of multimodality and promoted the fusion of multimodality and information. After constructing a systematic functional language, it is believed that there are nonfunctional language systems, such as actions, expressions, and colors. Under people's continuous research, it is generally accepted that these categories of symbols have certain special meanings. Their specific manifestation is that they not only play a certain supplementary role to language but also have relative independence. They are extended to the field of education. It is found that, in the classroom, the teachers and students can not only communicate and interact through language but also complete the process of teaching and learning through nonverbal communication [18]. In other words, the mode selection of classroom-teaching interaction is actually a process of building a systematic functional language system.

#### 3.2.3. Multimodal Concept

After having the foundation of social symbols and systematic functional language, people further put forward the theory of multimodality and systematized it. In daily life, some modal information that we come into contact with mainly includes text, image, video, and audio. The so-called multimodality is a modal expression that achieves a series of purposes by integrating or fusing two or more perceptible sensations. In today's multimodal development, various modal information is continuously blended. This has brought new developments to fields such as education and science and technology and has influenced and changed traditional processes. In the field of education, because of the diversity of teaching tasks, multimodality is quickly introduced into the process of teaching and classroom practice. Multimodality is also evolving in teaching and its practice.

### 3.3. Multimodal English Teaching

In the field of teaching, the fusion of multimodality has been overwhelming [19]. Especially in the process of English teaching, because of the particularity of English teaching, the trend of multimodal integration is stronger. From the perspective of a single modality, the English teaching process involves the combination and arrangement of multiple modalities, which fully demonstrates the characteristics of multimodal fusion. The first is the listening mode. If the listening information cannot be obtained from it in the English classroom, the communication in the classroom will be impossible. The second is the language modality. After obtaining the information through the listening modality, people must use the language modality to express certain expressions. Language is the basis of communication and, on this basis, people can interact with other modalities. The next step is to read. It involves the fusion of visual modalities and language modalities. Under the teacher's instruction, the students' vision and language continue to integrate and show certain interactive characteristics. Then the process of writing is an ingenious fusion between nonverbal modalities and kinesthetics [20]. Among them, in nonverbal communication, the teacher's expressions and gestures are the main modes of communication. After combining with the kinesthetic sense, students can feel the experience brought by the interaction more directly. The multimodal English teaching process framework is shown in Figure 4.

In the multimodal English teaching process, teachers often master a variety of modal means and combine a variety of modal teaching methods. In this process, students realize the interaction under various modalities through the choice of classroom interaction.

#### 3.3.1. Characteristics of English Teaching

English teaching has attracted much attention because of its language characteristics and interactive teaching characteristics. English teaching focuses on listening, speaking, reading, and writing. In this process, listening comes first. However, traditional English teaching is only from the perspective of single modal information, with blackboards and books as the main teaching materials. In the long-term teaching process, on the one hand, it is very difficult for students to learn English, and they often need a lot of self-awareness in the learning process. Because this learning method is boring, students cannot put in more enthusiasm for learning [21]. On the other hand, as a language course, talking about education without the color of the language will lead to the fragmentation of learning, so that students only know it but do not know why.

Therefore, it is imperative to incorporate a multimodal approach into English teaching. The reason is that teachers can assist foreign language teaching through body language teaching. Gestures, movements, facial expressions, and eye contact can convey different visual signals. The process of use of body language is actually a process of interaction. Appropriate body language can also stimulate students' visual senses, deepen students' understanding of English, and achieve interactive effects. In the process of continuous development of science and technology, the configuration of equipment and facilities in the field of teaching has become increasingly perfect from hardware resources to software resources. Teachers can make full use of classroom information technology and combine English teaching and computer teaching in the classroom. This is a teaching mode of single teaching by teachers, and, through the combination of multiple modes, the interest and richness of teaching can be realized. By triggering the students' auditory, visual, tactile, and other modalities, teachers can stimulate students' multiple reading abilities and English language application abilities. If the teaching materials are rich and the teaching methods are diversified, the classroom will change from single to diverse, from boring to active. This will also allow students to participate more actively in practice and improve their practical ability to apply English.

#### 3.3.2. Multimodal Teaching Principles in English Teaching

However, in the actual teaching field, the traditional teaching mode is relatively simple. It usually uses only one or two of the modal information types. In some classrooms, the use of modal information has reached two types. However, it is only a simple accumulation of modal information and does not fundamentally realize a multimodal teaching mode. In fact, there are many ways of multimodal teaching. Teachers can choose according to their own needs and the actual classroom activities. In the context of multimodal English teaching, there are usually several main teaching principles: subject adaptation, stage adaptation, and object adaptation [22].

*(1) Main Body Adaptation*. In the English teaching, classroom, teachers, and students are the main body in the teaching process. Therefore, in this process, the teacher should also mobilize a modal acceptance of the students while using a certain mode of teaching. Otherwise, students will gradually lose interest in the classroom because they cannot receive information from the teacher. Finally, I even lost interest in the subject of English. For example, in the listening process, teachers can choose more formal language materials according to the theme in the main class, such as celebrity interviews, current affairs analysis, and other materials. They can also broadcast more relaxed life phrases or dialogues during the introduction in class, allowing students to contact audio materials of various resources. However, at the same time, the selection of audio material should consider the English level of the students and match the actual ability of the students. The application of auditory modalities not only improves students' listening ability but also promotes students' speaking ability. The practice of spoken language requires students to convert auditory symbols into language symbols. This is then followed by language output through repeated imitation, which in turn achieves the fusion of multiple modalities.

*(2) Stage Adaptation.* At different stages of teaching, teachers should use different teaching methods. How multiple modalities can be presented in a classroom without conflict requires teachers to think carefully. For visual symbols, there are more opportunities to display visual symbols during the course. Therefore, teachers can enrich the classroom as long as they make appropriate arrangements when choosing. For hearing, the music material in English teaching can create a relaxed and pleasant atmosphere. It allows students to learn language in a pleasant and relaxed state of mind, which can transform learning into a kind of enjoyment. However, the songs used in teaching must have strict regulations, and songs cannot be used arbitrarily. Due to the different types of music, the meanings of the representations are also different. Playing the right song in the right scene helps to enhance the students' impression of the situation. However, the teacher must pay special attention to adjusting the sound to an appropriate level in time, so that the song cannot affect the classroom and the application of other modal symbols. The characteristics of foreign language network intervention teachers can infiltrate the network platform into the classroom teaching when they set up the curriculum. They recommend the characteristic foreign language teaching network to the students, so that the learners feel as if they have entered a website by browsing. Students are simultaneously impacted by multiple senses of sight, hearing, touch, and so on. When teachers conduct online teaching, they should make detailed comparisons according to each student's different English proficiency and different language needs. This helps students choose a foreign language website that suits their level and hobbies.

*(3) Object Adaptation*. In the process of English teaching, teachers and students are the main body of teaching. The teaching resources and content with curriculum and teaching content as the carrier become their objects together. In the actual process of teaching, teachers should combine teaching content reasonably and apply teaching resources and various media means to attract students' attention. For example, when showing sports, PPT teachers can use fast-paced music or English songs. As long as they control the volume a little, it will make the presentation of the picture fuller. Teachers can use soothing music as a background when introducing the cultural section. However, the choice of music must fit the theme. In addition to the application of audio files and music symbols, the stimulation of sound effects also has a stimulation method of auditory modality, which is the imitation of sound effects. For example, teachers can use different sound effects while showing pictures when explaining the difference between the sounds to the Chinese and Westerners. This can draw the attention of students and make the atmosphere of the classroom be more relaxing. Teachers can use the sound of wind chimes when explaining poems. Teachers explain the influence of nature on human beings and can play the sound effects of different scenes such as earthquakes, typhoons, rainstorms, and tsunamis. In this teaching process, teachers can also allow students to make independent guesses, which will further improve students' interest in learning.

#### 3.3.3. Classroom Interaction Based on Multimodal English Teaching

No matter what means teachers use in class, their main purpose is to interact with students, so that students can have an impression of the classroom and internalize the content of the course in their hearts. Therefore, in the process of teaching, how should teachers use multiple modes to form classroom interaction with students? We know that students mainly rely on books when learning, and the knowledge in books is the basis for students to learn. Then, in the process of classroom interaction, teachers need to pay attention to the fact that they must not be completely separated from the carrier of books. Although teachers should try to avoid the phenomenon of using only books in the class, they cannot completely leave books, because it will make students overwhelmed, without knowing what to focus on in class [23]. Therefore, the first visual symbol to be applied by teachers in teaching interaction is books. Then, teachers can let each student learn more about English through foreign language learning software under the condition of perfect hardware supporting equipment.

Secondly, teachers usually use blackboard writing in class and will generate language symbols, and the transmitted information will deepen students' impression of knowledge. In this process, blackboard writing itself is also a form of interaction. However, it is a kind of rigid interaction, and it cannot mobilize the interest of students. Therefore, when teachers are writing on the blackboard, appropriate blackboard writing and PPT conversion applications can help students avoid visual fatigue and strengthen interaction with students.

## 4. Artificial Neural Network Algorithm

In typical neural network calculations, the results are often affected by the number of neural network layers, the number of layers involved in the operation, and the number of units. To this end, we first add the nonlinear neuron parameter *n*, which infinitely approaches a constant *b* in the neural network, and its value range is [0, 10]. Concept *m* of the number of hidden layers of the neural network is introduced, and its related expressions are shown in the two following equations:

(1) $$\begin{array}{c} m=\sqrt{n+1}+b, \end{array}$$

(2) $$\begin{array}{c} m={\mathrm{lg}}^{b}. \end{array}$$

In the above equations, the nonlinear neuron parameter *n* is mainly affected by the number of layers and other factors. It can map the value in the range of [0,1]. In the following, we will mainly rely on this function to train the algorithm behavior.

At the same time, we use the activation function *S*, whose calculation is shown in formula (4).

(3) $$\begin{array}{c} n=\sqrt{b\times m}, \end{array}$$

(4) $$\begin{array}{c} S\left(n\right)=\frac{1}{1+e^{nx}}. \end{array}$$

In the operation, the input value and the actual value are somewhat different.

(5) $$\begin{array}{c} \lambda =\frac{1}{4}\sum_{i=1}^{n}{\left(e_{i}-y_{i}\right)}^{2}, \end{array}$$

where 1 and 2 are the expected and actual values of the input, respectively.

It is basically consistent with the variance principle. According to the relationship of the number of layers of the neural network, we can derive it.

(6) $$\begin{array}{c} \lambda =\frac{1}{4}\sum_{i=1}^{n}{\left(e_{i}-y_{i}\right)}^{2}=\frac{1}{4}\sum_{i=1}^{n}{\left(e_{i}-a\sum z_{m}\cdot z_{k}\right)}^{2}. \end{array}$$

After expanding the definition, we can obtain a correlation function between *λ* and the layer weights *z*_*m*_ and *z*_*k*_.

The goal is to continuously reduce the error. In this process, we found that we only need to find a small enough quantity; then if the error is also smaller than this small enough quantity, it can be shown that the error is small enough.

A sufficiently small amount of *δ* is introduced and suitable increments Δ*z*_*m*_ and Δz_k_ for the weights are found. Then, in the continuous iterative process, a minimum value can be obtained. By comparing it with a sufficiently small quantity, we can determine the local extent of these minima.

(7) $$\begin{array}{c} M_{a}=\sum_{m=1}^{n}x_{m}*z_{m},\\ N_{\text{a}}=\sum_{k=1}^{n}x_{k}*z_{k}. \end{array}$$

There are *m*=1,2,…, *n*, and *k*=1,2,…, *n*.

(8) $$\begin{array}{c} \Delta z_{m}=-\eta \frac{\partial \lambda }{\partial z_{m}},\\ \Delta z_{k}=-\eta \frac{\partial \lambda }{\partial z_{k}}. \end{array}$$

In the above equation, *η* represents the value of the increment, which is a range parameter of the scale coefficient property. By taking the partial derivative of it, we find that there is a minimum value in this formula.

(9) $$\begin{array}{c} ℑ=\left|\Delta z_{m,k}-\delta \right|, \end{array}$$

where *ℑ* is the difference between the minimum and small. A larger value indicates a larger difference, and a smaller value indicates that the two are closer.

(10) $$\begin{array}{c} \Phi ={ℑ}_{\max}-\frac{m\left({ℑ}_{\max}-{ℑ}_{\min}\right)}{m_{\max}}. \end{array}$$

In the above equation, *ℑ*_max_ is the maximum value of the difference weight, *ℑ*_min_ is the minimum value of the difference weight, m is the number of times of participating in the calculation, and m_max_ is the maximum number of calculations. According to different calculation times, we adjust the weight adaptively.

(11) $$\begin{array}{c} \Gamma ={ℑ}_{\max}-\frac{\left({ℑ}_{\max}-{ℑ}_{\min}\right)\times \left(m-m_{\min}\right)}{m_{avg}-m_{\min}},m\leq m_{\text{avg}},\\ \Gamma ={ℑ}_{\max},m>m_{avg}, \end{array}$$

where *m* is the number of computations at any time and *m*_avg_ is the average of all computations. After knowing the difference and the weight of the difference, we define a recursive callback function that follows the number of times. When the minimum number of computations as well as the learning speed is *σ*_min_ recursively, we can judge its efficiency.

(12) $$\begin{array}{c} \sigma_{\min}=\sum_{n=1}^{m}m_{avg},\left|m_{avg}-m_{\min}\right|\leq \left|m_{\max}-m_{avg}\right|. \end{array}$$

In unit time, the number of times and the efficiency of learning can be defined by the following formula:

(13) $$\begin{array}{c} \Omega \equiv \frac{1}{2}\sum_{u=1}^{m}\sqrt{Ra}+\frac{Ra}{2}\sum_{i=1}^{n_{h}}m_{i}z{\left(x_{i}\right)}^{2},\\ Ra=\sqrt{\frac{2}{m_{\max+}m_{\min}}}*Q. \end{array}$$

In the above equation, *Q* is an actual quantity parameter, which does not participate in the final calculation process and is a local variable.

Its meaning is described by the following formula:

(14) $$\begin{array}{c} Q=\left(m\_{\text{center}}_{n},m\_{\text{middle}}_{n}\right). \end{array}$$

In this process, the main purpose is to get the required variables.

After comparing the defined small enough quantities, we obtain the following formula using the number of network layers and calculations:

(15) $$\begin{array}{c} \varepsilon \left(m,n\right)=\sqrt{\sum_{n=1}^{m}{\left(a_{m}-b_{n}\right)}^{2}}, \end{array}$$

where *s* is the functional expression between the number of layers and the number of times.

(16) $$\begin{array}{c} s=\frac{\left[{\overset{\wedge }{m}}^{\left(1\right)}\left(n\right),s\right]}{\sum_{i=1}^{L}Ra_{n}}. \end{array}$$

At this point, all required variables and function expressions have been derived. To evaluate the accuracy of this calculation, we take a relatively small value *D* for it. We also perform the circle multiplication calculation and then enter the calculated result into the weight discriminant.

(17) $$\begin{array}{c} f_{n}=Q\left[D_{s}n\right]⊗\partial^{\left(i\right)}. \end{array}$$

The final precision value is double affected by the weight value *f* and the relatively small value *D*. The larger the value is, the more accurate the calculation is, and the smaller the value is, the larger the error is in the calculation.

(18) $$\begin{array}{c} \partial =\frac{f\left[{\overset{\wedge }{n}}^{\left(1\right)}\left(f\right),fn\right]}{\sum_{i=1}^{n}f\left[m^{\left(1\right)}\left(y\right),f_{i}\right]}. \end{array}$$

To preliminarily explore the retention rate of people's memory for the same knowledge point in a multimodal situation, we selected a specific knowledge point. It also made statistics on people's memory in different time periods. The results are shown in Table 1.

Table 1 shows that, under a single modality, people's memory retention is often less than 3 days and even only 10% of the original by the seventh day. The multimodal memory brings more profound and lasting memory and still has 30% retention on the seventh day.

After clarifying the effect of multimodality on people's memory, we decided to start from student achievement to explore the degree of influence of multimodality on student achievement.  Figure 5 shows the test scores of students at different stages.

Figure 5(a) shows that, at the beginning of the preliminary examination, the traditional teaching mode often helps students achieve good grades first. However, we found that the advantages brought by multimodal teaching have gradually emerged.  Figure 5(b) shows that, after mid-term, the multimodal teaching style continued its good effect on grades. The annual comprehensive score can reach 82, which far exceeds the two other teaching modes.

After witnessing the advantages of multimodality, we conducted group experiments by designing two experimental groups and one control group. Two of the experimental groups adopted the multimodal teaching method, respectively. However, the first experimental group used simple multimodal fusion, and the second used deepened multimodal fusion. The control group adopted the traditional teaching mode. After twelve weeks of teaching, we made statistics on the scores of these experimental groups. The results are shown in Table 2.

Table 2 shows that, compared with the control group, the performance of the experimental group was significantly better. Especially in terms of the number of people with scores below 60, the number of people in the experimental group was significantly lower than the number of people in the control group. We can see that the number of people in experimental group 2 is also much lower than that in group 1. In terms of high scores, although the number of people in group 1 has an obvious advantage, the final average score also explains the situation. The above data fully illustrate the advantages of the deepened multimodal fusion theory.

However, from the above data, we also found that although the experimental group has advantages under certain circumstances, the traditional teaching method is not without merit. Therefore, after having the foundation of multimodal teaching method, we introduce artificial neural network (ANN). It is also used to carry out different multimodal adaptations for different classrooms to achieve good results.

Before the start of the new course, we made simple statistics on the students' English abilities and a comprehensive assessment. The statistical results are shown in Table 3.

Table 3 shows that although students have been exposed to a certain mode of teaching, the overall average interest of students in English is still not high, and 33.1% of students expressed no interest. This shows that there are still many improvements in English classroom interaction and teaching under multimodality. Therefore, on the basis of the previous experiment, we introduced the characterization and comparison of several dimensions of classroom performance, interaction volume, grades, memory retention rate, classroom atmosphere, and students' enthusiasm. The results are shown in Figure 6.

Figure 6(a) shows that, after the multimodal deep fusion based on ANN, the students' performance and interaction in the English classroom have been greatly improved. This is nearly 10% higher than the traditional teaching model.  Figure 6(b) shows that the multimodal theory based on ANN can greatly mobilize the enthusiasm of the students, and it also helps to train the students' memory to a certain extent.

To study which modal teaching methods can be more favored by students and under which method, the students' classroom knowledge acquisition rate can be more guaranteed. We study the two previously mentioned questions. The results are shown in Tables 4 and 5.

Table 4 shows that the modality that most students are more willing to accept is the visual tactile modality. Among the students, 49.24% said they could get pleasure from it. This suggests that we can further study its knowledge acquisition in the same classroom using visual touch.

Table 5 shows that although visual touch is accepted by students because of visual and tactile impact, 32.42% of students are still unable to acquire effective knowledge in the classroom. This shows that the form that students like and hear is not necessarily the most efficient and effective form. From the table, we can also see that, based on the multimodal approach, 59.17% of the students can master most of the knowledge. However, at the same time, we also see that 5.11% of students still cannot acquire knowledge from it. Therefore, it is necessary for us to conduct related experiments on ANN-based multimodal teaching interaction.

With the support of the above data and the multimodal teaching interaction theory of ANN, we began to carry out different multimodal applications for different classrooms and student groups. Before this, we first apply ANN to predict the application of matching modalities of students under different classroom performance. At the same time, we also conduct modal matching experiments on these students.  Figure 7 shows a comparison of the predictions with and without ANN-based predictions and the measured results.

Figure 7(a) shows that, without introducing ANN prediction, there is still a big difference between the prediction results and the practical test results, especially in the third and fifth experiments.  Figure 7(b) shows that the fit between the predictions and the actual results is much stronger after introducing the ANN's prediction.

From the above data, we cannot clearly see the gap between the forecast and the actual data. After estimating the difference between the two, the relative errors of the above two prediction results are shown in Figure 8.

Figure 8(a) shows that, without introducing ANN, the relative error between the measured and predicted data fluctuates greatly, with a peak of more than 10%.  Figure 8(b) shows that, after the introduction of the ANN, the difference between its predictions and the actual data is significantly reduced.

Although the peak value has reached 5% in some experiments, the accuracy is relatively guaranteed. After the targeted use of multimodal English teaching and interaction, we reevaluated students' abilities and interests in English. The results are shown in Table 6.

The results in Table 6 show that, after the multimodal English teaching interaction based on ANN, the students' comprehensive interest in English is as high as 81.9%. At the same time, the students' interest in English listening, speaking, reading, and writing has also been improved to a certain extent.

Interest is the best teacher. After students are full of interest in English teaching, we have carried out a series of multimodal English teaching interactions based on ANN.  Table 7 shows the students' test scores after the course.

Table 7 shows that, by comparison with the previous control group and experimental group, the students' English performance after ANN has been greatly improved. Its average score can reach 85.17, which is much higher than the previous 78.31.

## 5. Discussion

In a multimodal environment, the integration of English teaching and multimodality can readjust and upgrade the English teaching mode. In this process, the combination of multimodality and artificial neural network can effectively strengthen the interaction between teachers and students and improve the interaction rate of the classroom. It changes the traditional English classroom from boring to active and enhances students' interest. In the teaching process, as long as the teacher follows the modal theory in an orderly manner and combines the prediction of ANN, the modal teaching can be beneficial without any harm, which will improve the students' reading, listening, speaking, and communication abilities. In the system construction of multimodal English teaching and classroom interaction, English teaching has gradually realized an integrated multimodal interactive classroom, which provides a good reference for the adjustment of teaching modes in other disciplines. At the same time, teachers should also take the multimodal theory based on artificial neural network as a new research field of English teaching method. It is necessary to pay full attention to the influence of the multimodal teaching interaction model under the artificial neural network on the cultivation of English interaction ability.

## 6. Conclusion

This paper studies an interactive method of multimodal English teaching based on artificial neural networks. It also discusses the fusion theory of different modalities in the context of artificial neural networks. This reveals the necessity of applying artificial neural networks and multimodal theory to English teaching interaction from both theoretical and practical aspects. In this paper, the multimodal English teaching interaction theory based on artificial neural network has a certain role in improving the interaction ability of teachers and students, but this research also has some shortcomings. First of all, the sample data of the experiment in this paper is valid, and the research objects limit the depiction of the whole picture, so there may be insufficient representativeness. Second, this research lacks the ability to combine theoretical foundations with practical English teaching more deeply, which affects the breadth and depth of interactive research on multimodal English teaching. Finally, this paper does not exclude the interference objects in the experiment. In the future, the research depth of this field needs to be further explored.

## Figures and Tables

**Figure 1:** Neuron structure.

**Figure 2:** Artificial neural network and neurons.

**Figure 3:** Application areas of artificial neural network.

**Figure 4:** Multimodal English teaching process framework.

**Figure 5:** Test scores of students at different stages.

**Figure 6:** Multimodal deep integration of classroom interaction and efficiency based on ANN.

**Figure 7:** Student matching modal prediction under different classroom performance.

**Figure 8:** Student matching modal prediction error under different classroom performance.

**Table 1:** Students' memory of the same knowledge.

Sense organs	Time and memory retention		
	Three hours later (%)	Three days later (%)	Seven days later (%)
Hearing only	55	20	11
Only use vision	60	19	9
Touch only	50	39	12
Multimodal	75	45	30

**Table 2:** The results of the experimental group and the control group.

Score class	Below 60 points	60–70 points	70–80 points	80–90 points	Average scores
Experiment 1	8	16	30	11	77.96
Experiment 2	5	15	35	10	78.31
Control class	12	13	34	6	70.23

**Table 3:** Students' interest in English.

Interested	English reading (%)	English writing (%)	English listening (%)	English expression (%)	English comprehensive course (%)
Yes	31.7	29.6	29.1	32.4	31.7
No	41.2	20.3	37.2	39.4	33.1
I cannot say	27.1	50.1	33.7	28.2	34.2

**Table 4:** Teaching modes favored by students.

Options	Hearing and speech modalities (%)	Visual and tactile modalities (%)	Language and image modalities (%)
Very large	9.57	28.97	18.97
Larger	32.14	49.24	39.24
A little bit of impact	48.29	21.79	41.79
No	7.21	9.39	6.30

**Table 5:** The knowledge absorption rate of students under various teaching modes.

Options	Hearing modalities (%)	Visual modalities (%)	Language modalities (%)	Multimodal (%)
Get all	4.57	2.98	6.12	15.22
Get most	39.14	39.24	31.76	59.17
Get a little	38.29	21.76	30.66	27.26
Get nothing	20.90	32.42	14.34	5.11

**Table 6:** Students' comprehensive interest in English.

Interested	English reading (%)	English writing (%)	English listening (%)	English expression (%)	English comprehensive course
Yes	61.7	59.8	69.1	72.3	81.9%
No	10.6	20.1	17.2	9.4	3.9%
I cannot say	27.7	20.1	13.7	18.3	14.2

**Table 7:** Students' test scores.

Scores group	Below 60 points	60–70 points	70–80 points	80–90 points	Average scores
Previous grades	12	13	34	6	70.23
After the ANN	2	23	30	10	85.17
Average score	7	18	32	8	75.25

## Data Availability

The data underlying the results presented in the study are available within the article.
